# Investigation of management of international education considering sustainable medical tourism and entrepreneurship

This article has been retracted.

**DOI:** 10.1016/j.heliyon.2022.e12691

**Published:** 2023-01-07

**Authors:** Aoqi Xu, Seyed Abdolhassan Johari, Amir Hossein Khademolomoom, Mohsen Tavakoli Khabaz, Rajabov Sherzod Umurzoqovich, Saeed Hosseini, D.T. Semiromi

**Affiliations:** a School of Economics, Fujian Normal University, Fuzhou 350007, China; b Master of Business Administration, Management Faculty, Tehran University, Iran; c Institute of Social Sciences, University of Mediterraniean Karpasia, Şht.M. Ruso Cad. No. 79 Belyaka Sk, North Cyprus via Mersin 10, Lefkoşa, Turkey; d Faculty of Management, Kharazmi University, Tehran, Iran; e The Head of the Department of Quality Control of Education, Tashkent Institute of Finance, Tashkent, Uzbekistan; f Faculty of Management, Islamic Azad University, Sanandaj Branch, Sanandaj, Iran; g Mechanical Engineering Department, Islamic Azad University, Isfahan, Iran

**Keywords:** Management, Communication technology, Sustainability, Medical tourism, Entrepreneurship

## Abstract

Medical tourism leads to development of economic resources for many countries. This method of tourism has become common in most countries of the world which is one of the dimensions of tourism for development like metal industry or sport industry. The stability and dynamism of country's economy help the development of ecotourism. Furthermore, medical tourism with economic consequences can have significant environmental effects. For this purpose, this research was done to study and evaluate the factors affecting the development of medical tourism in developing countries. The approach governing this research is developmental, and the research method is descriptive and analytical. A multivariate regression test was used to analyze the hypotheses of research, and statistical analysis was conducted using SPSS 19.0 software. The ecotourism and economic management can have a global or local roles as suitable tools for sustainable tourism. Ecotourism is often not properly oriented and mainly defined in such a way that the practitioners are far from the declared standards to achieve and succeed in the sustainability process. The current research is descriptive-explanatory which compiled using library documents. The analysis of the path of above factors shows that all factors of price, quality, facilities, and information and communication technology directly and indirectly play a significant role to enhance the medical tourism.

## 1 Introduction

Today, the subject of management plays an irreplaceable role in various fields such as risk management, system management, resource management, project management, thermal management, etc., and researchers have done a lot of research on it [[1], [2], [3], [4], [5], [6], [7], [8], [9], [10]]. The expansion of tourism industry causes the migration of students from other countries to another country and improves the tourism situation [[11], [12], [13], [14]]. To increase the capacities of medical tourism, these students can be good ambassadors for this industry for their fellow citizens and countrymen. “Transformation and Development” to the purpose of this transformation and development is to emphasize the locality, strengthen normality, cultivate practical abilities and serve local economic and social growth [[15], [16], [17], [18], [19]], enrich the theoretical research of higher education and compensate for the lack of research on the development of new conventional colleges. Therefore, further guidance and the standardization of school administration behavior are needed [[20], [21], [22]]. Nowadays, the medical tourism industry is ranked third due to income generation and countries have made many efforts to develop the state of this industry. Many countries are developing programs for excellence, earning, and creating jobs via the medical tourism industry [23–27]. As the largest commercial sector in the world, tourism has created the employment for more than two hundred million people and accounted for more than 8% of world's jobs. It is one of the five main sources of foreign exchange products in developed and developing countries [16–19]. Foreign income is considered the first income source in 50 countries, including Italy, France, Iran and Australia. Tourism is considered the primary source of foreign exchange production for more than 38% of developing countries and the main part of foreign exchange for 1.8% of the poorest countries [19–24]. Apart from the financial benefits of tourism, tourism as a multi-valued issue is one of the important ways to achieve Sustainable Development (SD) which is an inexhaustible resource with minimal environmental destructive effects [[24], [25], [26], [27], [28]]. The medical tourism industry related to hotels, airlines, and welfare-entertainment activities [[29], [30], [31], [32], [33], [34], [35], [36]]. The medical tourism industry can easily find coordination with relevant business, such as hospitals, insurance companies, and newly established travel agencies [[36], [37], [38], [39], [40], [41], [42], [43], [44], [45], [46], [47]]. The travels of tourist made to obtain health issues are growing to Eastern Asian countries. Many of these countries have proper electrical devices and facilities which have international medical, health and wellness standards. It is high quality of service provision within the capacity of Eastern Asian countries. Medical tourism can provide the basis for the country's future growth, and it follows global economic crisis. In this research, the type of communication and interaction between the employees of medical centers and tourists who migrate to developed and semi-developed countries for medical treatment have been investigated.

## 2 Research methodology

### 2.1 Conceptual model of medical tourism research

The research method is descriptive-analytical which considers studying the effects of tourism to create environmental pollution, the technique of collecting information is the overview of the library, and the research method is descriptive-analytical. The effects of tourism in creating environmental pollution, collecting information in the form of a library, review, and different sources were used to process the data. Selecting the environmental indicators is directly related to the environmental situation and the goals and activities of tourism area. In general, several main criteria can be considered to select these indicators based on indicator connection with the selected topic, the possibility of obtaining and analyzing the required information, reliability and validity of information for users of these information, transparency, and comprehensibility of these data for users and comparability over time and across regions needs to be studied. In tourism field, among the factors which are involved in selecting the environmental indicators, following indicator can be mentioned as an environmental, political, social, cultural, economic conditions, technical issues, the presence of tourism infrastructure, the type of tourism services and activities, the number of tourists in the region, and the place of tourism in the local economy regional [48–52]. Three main criteria and bases used in OECD is the relationship with the policy which an environmental indicator should show an example of environmental conditions, pressures on the environment or society's reactions.

### 2.2 Analytical accuracy

An environmental indicator should be well founded from a theoretical point of view in scientific and practical formats to have the ability to communicate with economic models for forecasting the situation and information systems [53–55]. The determined model should be able to measure the necessary data to support the index at a reasonable cost/benefit ratio. Fig. 1 indicates how these three factors are interrelated and significantly affect upon each other. To review the results and descriptive statistics via the interviews with university professors and experts in the fields of economy, culture, and information and communication technology, it was confirmed the proposed model. A multivariate regression test was used to analyze the hypotheses of research, and statistical analysis was performed using SPSS 19.0 software. Fig. 1 shows the management triangle in tourism which is the most important factors, such as place, host community, and visitor that can have a significant effect on the connection of all three important parts of external effects. In the examination of Fig. 2, which was done by the researchers, it was found that this simple triangle can be of great help for managerial decision-making in medical tourism. It indicates that the place of tourism activity is the main part of tourism. It is found that many researchers' efforts were made to link the tourist destination with the productive environment of tourism. Fig. 2 shows the relationship among the areas formed for tourism and the destination areas which tourists are passing through. The effective factors on the tourism process include political, social, cultural, economic, and environmental. This tourism system was identified as a manufactured spatial. Effective factors in tourism development among the factors that can develop the country's tourism industry is using effective marketing tools and parameters. One of the weaknesses of tourism in Islamic countries like Oman, Iran and Iraq is the lack of extensive advertising to attract the target market. Economic factors are considered from two points of view.

**Fig. 1:** The triangle of three major components in tourism management (Adapted from ETB, 1991.).

**Fig. 2:** The tourism system: a spatial construct.

## 3 Results

### 3.1 Tourism development analysis

Social and cultural factors directly affect the development of tourism in the form of population growth and urbanization [56–64]. Reducing working hours and increasing the duration of vacations, and visiting different and unknown places are effective in developing tourism. Tourism develops profitable local industries and prospers the region at the local level via the construction of hotels, restaurants, transportation systems, handicrafts, local gifts, and guide services. Tourism attracts foreign currency, and thus helps local and regional economies [49]. Tourism has diversified the local economy, especially in rural areas, because agricultural jobs may be concentrated which can cause diversity and scope of employment. Tourism contributes to the local economy by creating demand for agricultural products and injecting capital. Tourism improves the transportation network, communication, and infrastructure factors and benefits local people. Tourism causes beneficial exploitation of some lands considered marginal lands for farmers, and the areas of a large part of the land to remain with natural cover [65–68]. Tourism has caused the transfer of cultures to each other and provides the field of communication in the global dimension and improves the level of people's understanding of each other's culture. As tourism is well managed, it can be considered a mechanism for self-management of natural-cultural environments as a tool to protect natural heritage. Tourism provides suitable resort facilities which can be used by local communities, as well as domestic and foreign visitors [69–82]. Regarding its tangible achievements, tourism is a means to convince government officials and the general public about the importance of protecting natural areas. These benefits show themselves more prominently when the protected areas devoted to tourism are least useful for agriculture. These benefits may become more valuable as they reduce access to other resort areas. The values and importance of employment-generating tourism in the world have generated millions direct and indirect job opportunities accounted for 10% of total global employment [61–81]. According to the surveys, five new jobs are created for each tourist arrival, including tour guides, the employees of tourist and tourism companies, the employees of hotels, guesthouses, restaurants, supermarkets, translators, training staff for managers and planners. The global growth trend in the tourism field for the countries located in South America with more than 10% was in the top row of the world growth table in 2011, followed by Europe with more than 6% as shown in Table 1. South Asia and Southeast Asia with more than 9% of growth have benefited from increased regional markets, while competitive growth in Northeast Asia weakened by more than 4%. African countries still maintain their 50 million tourists; however, North African countries have witnessed a 12% decline.

**Table 1:** Prediction of medical tourism till 2020 (million person).

Country	2010	2020
**Europe**	527	717
**West Asia**	23	438
**America**	195	284
**Africa**	46	75
**Middle east**	37	69
**East Asia**	11	19
**Total**	1.740	1.206

The number of international tourists has reached a new record despite facing the current challenges and conditions. The reason for this growth directly provided five percent of total global GDP and six percent of the total world exports. Therefore, various definitions of sustainable tourism were provided. A type of tourism which can be maintained in the long term, because it leads to a net profit from the social, economic, natural, and cultural environments of tourism area. A type of tourism does not endanger the cultural, social, economic or environmental integrity of the tourist destination in the long term. Sustainable tourism is considered a leader in the management of all resources. Therefore, economic, social and aesthetic requirement can be met, along with maintaining cultural integrity, basic ecological processes, biodiversity, and life support systems. This type of tourism should not be confused with other types, especially ecotourism.

### 3.2 Tourism and sustainable development

SD means improving the quality of human life by supporting the capacity to maintain ecosystems by providing strategies and tools that can respond to human requirements. Since SD is discussed in social, economic, cultural, political, and ecological dimensions and all mentioned cases are considered in developing tourism industry; therefore, taking advantage of this point of view in the development of tourism industry is of particular importance. Some examples of positive environmental, cultural, social, economic, and political effects of tourism in the direction of SD are mentioned in following paragraph. Tourism and environmental pollution are a phenomenon which includes many activities cause harmful effects on our environment. The water pollution issues by sewage, garbage production by tourists, environmental damage resulting from land destruction, air and noise pollution caused by the movement of airplanes are among these effects. Traveling to different regions requires more infrastructure development, such as road construction, building hotels and similar facilities that the implementation of each one may lead to more exploitation of natural resources, as well as pollution of water, air and the environment as a whole. Furthermore, the growth of tourism causes an increase in energy demand and usually involves environmental destruction. The disturbance of ecological balance and order of the environment, change of using lands especially agricultural land, reduction of aesthetic, architectural values, loss of landscapes and urban development are other complications of tourism development. Selection and design of the most suitable water and sewage systems, providing technical solutions for solid waste disposal, technical solutions for air and noise pollution, placement of buildings, structures and facilities, providing solutions regarding the selection, design and management of national parks and compliance with design standards, construction, control and development are among the topics discussed in this topic. In different regions of the world, tourism development is associated with environmental protection in which governments emphasize these issues. Tourism can endanger the natural environment with a negative effect, such as noise and visual pollution. Natural attractions can be endangered by improper or excessive use [[50], [51], [52], [53], [54], [55], [56], [57]].

### 3.3 Proposed causal model

The construction of non-conventional constructions for tourists can change natural scenery and its appearance. By surveying various studies which were comprehensively conducted, from sources, such as books, research articles, conferences, theses, research projects, etc., direct effect of factors such as quality of medical and tourist services, medical facilities and communication technology on medical tourism in different world regions was studied. It is quite evident that the indirect effects of factors mentioned in conducted research are effective. A conceptual model was used for medical tourism to examine the presented model to what extent it can identify the direct and indirect effects of above factors on the development of medical tourism [58,59]. It was found that facilities and infrastructure highly affect the development of medical tourism. The indirect effects of other factors that were not studied in previous researches via the interviews were confirmed with university professors and experts in the fields of economy, culture, and communication technology and included in proposed model. Fig. 3 shows proposed model for developing medical tourism based on the relationships between research variables and developing medical tourism. It shows three factors of price and quality which cause the development of medical tourism, and the culture is in the middle of this relationship, and information and communication technology, facilities, facilities, and infrastructure are all directly related to culture. Based on available data in following Table 1, and relying on R^2^ values, 58% of the changes in the dependent variable are directly explained by above variables. As can be seen, the regression model with above 5 variables can explain 0.58 of the changes in the medical tourism development variable. Therefore, 0.42 of the changes in the dependent variable are explained by other variables which were not considered. Many hospitals in popular destinations provide staff at the level of hospitals in developed countries and pay for themselves. Considering the similarity of cost and treatment levels of developing countries and medical tourism destinations, many American and European doctors are immigrating to these countries, and the presence of European doctors in Southeast Asian medical tourism areas such as Singapore and Thailand. In the countries like Ukraine, these years are considered normal.

**Fig. 3:** Proposed model regarding the relationships between research variables and the development of medical tourism.

## 4 Discussion

Based on beta coefficients, the price variable of medical tourism services has a negative and inverse relationship with the variable of development in this area. An increasing rate of medical services and tourism leads to less development of medical tourism and vice versa. Moreover, the qualitative variables of medical tourism services, cultural, facilities, medical and tourist device, information and communication technology have a suitable relationship with development subject. Medical tourism is an international phenomenon with personal travel that tourists travel to reach medical services in terms of high costs, long waiting times, the lack of insurance, limited use of services and lack of access to medical services at the destination. This industry is now considered one of the most prosperous tourism markets in the world with an annual income of billion dollars and an annual growth of 21% [35–49]. Creating and promoting medical tourism in tourism has social and economic dimensions [50–54]. Medical tourism as a part of tourism industry was significantly promoted by many governments in post-industrial world, and many countries are currently establishing practical and legal programs to provide services. The entry of investors and entrepreneurs in this field has made the entry of private sector funds and the construction of specialized hospitals with modern equipment to help a lot in the treatment of certain diseases, including types of cancer and diabetes [55–61]. Although these centers could not attract clients from outside their native region due to current costs, they have greatly contributed to the rapid treatment of patients [62–69]. Creating cheap banking facilities and discounts and tax exemptions may make these investors more interested in this field. The suggestions based on the obtained results and the interpretation of the main goal of this study for developing medical tourism in developing countries are presented, which includes the costs of medical and tourist services should be clear, transparent and competitive so that the patients are aware of the cost of services compared to the costs of other countries [60–68]. Since the cost of performing these surgeries is very high in some countries, if another country pays less for the treatment, it can become an attractive and economical option. To attract health tourists, health tourism areas with fully equipped medical centers are considered in each country. In medical tourism industry, the cost parameter, along with time is one of the most important concerns. Another important benefit of medical tourism is the provision of urgent medical services in a short period of time. Medical tourism is an effective solution for the patients whose health needs immediate attention and who cannot receive such medical care in domestic hospitals in their own country [68–78].

### 4.1 Medical tourism risk

Medical tourism includes a series of risks which usually the patients in their own country face such risks less. The countries, such as India, South Africa, or Taiwan have many people suffering from epidemic diseases, such as hepatitis, malaria, typhoid or various types of influenza. Despite the compliance of standards by doctors, being in such environments increases the possibility of getting infected with these diseases. Diagnosing the quality of doctor's work is a kind of problem. The doctor may not have enough knowledge, and legal follow-up in a foreign country may not be possible easily if there is no problem. Therefore, tourists need to consider all aspects for some reason, the patient's condition worsens during the treatment and the doctor determines that longer procedures are needed. Besides, the costs may be several times higher than the expected cost. It is important to have someone from family or friends with patients, therefore the cost of hoteling increases. In fact, having a companion means twice the cost of flights, hotels, etc. The quality of services after surgery is varied in different countries, which may not match people's expectations. Similarly, as the patient intends to return to his/her country after the surgery, there is a possibility of aggravating the complications after the operation during long air trips and frequent relocations. According to research conducted in Norway, the worst part of medical tourism is the patient's pains and problems during his/her return to his/her country. Another problem of medical tourism is the popularization of illegal buying and selling of body organs, which is very common in populous countries, such as India and China. The present laws in the tourism industry and general planning and the basic components of the education system of countries have a significant effect on improving the economic situation of the tourism industry and similar areas. Studying the environmental conditions and problems in this industry should be considered, for example, visual pollution can occur via the installation of many billboards that make the city look industrial and stressful for tourism. Following the increase in population and pressure on natural resources, tourism has adverse effects on the environment. The issues, such as soil erosion, loss of swamps, destruction of wetland habitats, drying up or contamination of underground water and jeopardizing health and safety in terms of inadequate waste and sewage disposal networks threaten human societies. SD as a guide for management and planning of all resources can be a suitable option in order to meet the economic and social needs of tourism host cities.

### 4.2 General observation

Therefore, enhancing the environmental management of tourism facilities to reduce its damage is the first step to achieve the goals of the SD of tourism, especially in health tourism, because the patient needs trust and peace. The factor that causes the patient to use his country and city for medical tourism is to create peace and trust in the equipment and sometimes the quality of health services. WTO reports were many discussions about the causes of environmental problems, but it is still not possible to definitively analyze and study these causes, even among those who doubt about these problems. However, it is certain that the environment is changing due to human activities and facing catastrophic consequences. Keeping the price low is one of the main success factors of medical tourism. For example, the most common reason Americans travel for medical care is cheap prices in other countries. Nowadays, using smart city services with high reliability, it is possible to attract tourists and expand their advertisements [63]. Several studies conducted showed that tourism experience has always been a hot topic in research field in a way that it has its interpretation for any type of tourism with any conditions [64]. Using smart technology, the changes can be made in present models in tourism and the way of consumption and create better facilitation for travelers [65]. Using intelligent systems, these systems are fundamentally able to control the improvement effect using an appropriate assumption [66]. By examining the articles in this field, it was determined why tourism prefers a geographic region over the size of regions [67]. In the conditions of today's century, it is very important to investigate and study the quality and behavior of tourism in the development of cities [68]. The treatment of different and new diseases caused by nerve problems is progressing greatly via medical tourism because medical tourism centers have already treated these special diseases and built appropriate treatment conditions [69]. Time and speed are very important factors in medical tourism. For instance, Canadian patient waiting time for some surgeries is about 26 weeks on the waiting list. While the same operation can be done in Singapore, Taiwan, or India within a few days after the patient's admission which highly affect the medical tourism development [70–75]. Many reasons make people travel for treatment outside their country of residence, such as frustration with treatment in the country, lack of access to medical and therapeutic care at the right time and cost, and insufficient income to cover the costs. Local health services include high quality of medical care and treatment in developing countries, the desire to receive medical care far from the usual place, not having a waiting list, increasing popularity of health and medical services abroad, and access to the latest technologies [[71], [72], [73], [74], [75], [76], [77]]. Considering different positive effects of medical tourism on the country's economy, doctors and nurses find more motivation to stay and work in their country via health tourism. Recent surveys show that with the results obtained from the interviewees in the field of medical tourism and facilities on the environmental and social dimensions of sustainability, they have not predicted clear results and future for this field. Furthermore, most of them have introduced the possibilities of medical tourism on social dimension and attracting local doctors, integrating advanced technology and generating income for other sectors (transportation, accommodation, travel agencies), and not having elite specialists as the reasons for the weakness of this field. None of the interviewees mentioned gender equality, poverty and cultural awareness [75–79]. Several works by other researchers showed the lack of the same point of view of the interviewers in the field of medical tourism and the lack of social sustainability, which is consistent with the observations of researchers, such as Prayag et al. [80], Jones et al. [81] and Santos et al. [82]. Many studies showed that it defines the sustainability perception of hotel stakeholders [79–81]. Researchers in 2004 introduced that the most important factors hindering the development of this industry in India are the lack of initiative of government, the lack of coordination of elements, an accreditation mechanism for hospitals, and an integrated price and standard policy in hospitals [82].

## 5 Conclusion

SD in the medical tourism industry is the most suitable approach in this field, and ecological and socio-economic factor can be simultaneously developed in a society. In many advanced countries, tourism has a special place and is considered a very important resource in the economy of that country. Regarding the development of tourism and its sustainable estimation, special attention should be paid to the economic benefits and social consequences of tourism. The tourism industry includes various activities which is directly and indirectly related to economic, social, and cultural sectors. Therefore, one of the basic factors in the development and transformation of tourism sector is the comprehensive examination of positive and negative effects and a regional view of tourism development. Moreover, planning at all academic and even industrial levels is needed to achieve success in tourism development. Tourism development may not be successful without academic and educational planning, and it may cause social, economic and environmental problems for the host community. Thus, examining the environmental effects is very important. For the SD of tourism and planning in this field, the organizations that benefit from the advantages of tourism should be more involved and allocate part of their income from tourism to the well-being and provision of services to tourists to play an effective role in SD. Following the increase in population and pressure on natural resources, the issue of tourism leaves adverse effects on the environment. The issues, such as soil erosion, changing the coastline, destruction of coastal habitats, drying up or contamination of groundwater, and jeopardizing health and safety in terms of inadequate waste and sewage disposal networks threaten human societies. The best way to solve this problem is to use SD, which is considered a guide to manage all resources.

## Funding statement

This work was financially supported by the project of the 10.13039/501100001809National Social Science Foundation (21BJL052; 20BJY020; 20BJL127; 19BJY090); the 2018 Fujian Social Science Planning Project (FJ2018B067). The Planning Fund Project of Humanities and Social Sciences Research of the Ministry of Education in 2019 (19YJA790102).

## Author contribution statement

Aoqi Xu; Seyed Abdolhassan Johari; Amirhossein Khademolomoom; Mohsen Tavakoli Khabaz; Rajabov Sherzod Umurzoqovich; Saeed Hosseini; Davood Toghraie: Conceived and designed the experiments; Performed the experiments; Analyzed and interpreted the data; Contributed reagents, materials, analysis tools or data; Wrote the paper.

## Data availability statement

No data was used for the research described in the article.

## Declaration of competing interest

The authors declare that they have no known competing financial interests or personal relationships that could have appeared to influence the work reported in this paper.
